# Assessment of antioxidant, anticancer and antimicrobial activity of two vegetable species of *Amaranthus* in Bangladesh

**DOI:** 10.1186/s12906-016-1130-0

**Published:** 2016-05-31

**Authors:** M. Abdulla Al-Mamun, Jamiatul Husna, Masuda Khatun, Rubait Hasan, M. Kamruzzaman, K. M. F. Hoque, M. Abu Reza, Z. Ferdousi

**Affiliations:** Protein Science Lab, Department of Genetic Engineering and Biotechnology, University of Rajshahi, Rajshahi, 6205 Bangladesh

**Keywords:** *Amaranthus*, Anticancer, Antimicrobial, Antioxidant, Apoptosis, EAC cells, Lectin and mice

## Abstract

**Background:**

*Amaranthus* (*Amaranthaceae*) has previously been reported to possess different bioactive phytochemicals including phenols, tannins and flavonoids. The current study was designed to evaluate the antioxidant, anti-proliferative and antimicrobial activity of stem and seed extracts of *Amaranthus lividus* (AL) and *Amaranthus hybridus* (AH), respectively.

**Methods:**

Antioxidant activity of methanol extract was assessed by DPPH radical scavenging assay. Determination of lectin activity of *Amaranthus* extract was carried out using hemagglutination assay on mouse blood. A total of thirty six Swiss albino mice containing Ehrlich’s ascites carcinoma (EAC) cells were treated with AL and AH extract at 25, 50 and 100 μg/ml/day/mouse for six days. Growth inhibitory activity was determined by haemocytometer counting of EAC cells using trypan blue dye and DAPI (4΄,6-diamidino-2-phenylindole) staining was used to assess apoptotic cells. Gene amplification study was conducted to observe the expression pattern of p53, Bax, Bcl-2 and caspase-3 mRNA using PCR (polymer chain reaction) technique. In vitro susceptibility of five pathogenic bacteria including *Escherichia coli, Pseudomonas aeruginosa*, *Bacillus subtilis, Salmonella typhi* and *Staphylococcus aureus* was detected using disk diffusion assay.

**Results:**

The radical scavenging assay indicated that AH and AL possesses potent antioxidant potential, exhibiting IC_50_ value of 28 ± 1.5 and 93 ± 3.23 μg/ml, respectively. Hemagglutination assay revealed that AH and AL agglutinated mice blood at 1.565 and 3.125 μg/wall, respectively. Administration of AH and AL extract led to 45 and 43 % growth inhibition of EAC cells, respectively at 100 μg/ml with marked features of apoptosis including cell shrinkage, condensation of cytoplasm and aggregation of apoptotic bodies etc. Up-regulation of p53, Bax and caspase-3 and down-regulation of Bcl-2 mRNA in *Amaranthus* treated mice indicated mitochondria mediated apoptosis of EAC cells in comparison with control. None of the bacterial species showed susceptibility to the extract of both the *Amaranthus* species.

**Conclusion:**

Our current findings suggest that both of the *Amaranthus* species have strong antioxidant, lectin and anti-proliferative activity on EAC cells. The current anticancer potential was observed due mainly to the mitochondria mediated apoptosis of EAC cells.

## Background

Cancer is the prevalent worldwide fatal disease with high rate of mortality and morbidity. In 2012, an estimated 14.1 million new cases of cancer occurred and 8.2 million deaths worldwide [1]. The poor clinical outcomes against the cancer types are mainly attributed to the diversity in characteristics of specific cancer type and resistance to programmed cell death due to loss of the cellular ability to regulate the cell cycle negatively which allows the cells to proliferate abnormally and developing cancer [2]. Elevated level of reactive oxygen species (ROS), produced from both extracellular (irradiation) and intracellular (electron transport chain in mitochondria) sources reacts with DNA and cellular proteins, resulting base alteration, unstable genomes and genetic changes [3]. These types of molecular modifications lead to alter the normal apoptotic signaling machinery followed by uncontrolled cell proliferation and tumor formation [4]. Antioxidants are the biochemical constituents, produced in the body in insufficient amount, requiring external supply mainly from diet and having capacity to eliminate free radicals by neutralizing, quenching, reducing or through decomposing [5]. A plethora of studies suggest that there is strong correlation between the imbalance of antioxidant level and the development of several chronic diseases including cancer [6], neurologic disorder [7], cardiovascular disease [8] and age related disease [9].

Natural products are considered traditionally as the rich source of phytochemicals with various bio-structures and potent bioactivities against a number of diseases including cancer and infectious diseases. More than 80 % of the total world’s population relies on herbal medicine to meet their primary health care needs [10]. Current pharmaceutical industries are depending to a larger extant on natural products as a source of potential drug candidates as statistics show that over 60 % of the current anticancer drugs are related with herbal product as their origin [11]. A range of studies have confirmed that plant derived materials possess potential bioactive compounds and exhibiting considerable antimicrobial [12], anticancer [13] and antioxidant [14] activity. Generally, phytochemicals exert their anti-proliferative role by modulating the apoptotic signaling pathways in cancer cells which is considered as the key event in the antitumor activity [15]. Though the chemotherapeutic drugs are the good option to remedy from cancer, but they are not devoid of some drawbacks such as severe side effects and drug resistance etc. Therefore, exploring novel plant derived bioactive agents having anticancer and antimicrobial potential would contribute to manage the drug resistance and toxicity.

*Amaranthus* belonging to the family of *Amaranthaceae*, having approximately 60 species, distributed throughout the tropical and subtropical countries including Bangladesh. Different edible species of *Amaranthus* are being consumed widely as leafy vegetable across the world due mainly to its lower price and rich source of protein, carotenoids, vitamin C, dietary fiber [16] and minerals such as calcium, iron, zinc and magnesium [17]. Several species of *Amaranthus* have been reported to contain various bioactive phytochemicals such as carotenoids, ascorbic acid, flavonoids and phenolic acids etc [18]. *Amaranthus* has well been documented to possess important pharmacological properties including anticancer [19, 20], anti-inflammatory [21] and antioxidant activity [18]. Among the *Amaranthus* species, AL (locally known Sobuj data) and AH (locally known Lal data*)* are prevalent in South East Asian territory and are being consumed by all classes of people especially lower income group. Both of the species are 100-300 cm in height and grow annually as an erect, monoecious herb with several branches (30-60 cm) containing flower as terminal whorls.

In spite of having potent anticancer role of different *Amaranthus* species [19, 20] as well as the popular use of AL and AH in Bangladesh, there are no sufficient reports regarding the anticancer and lectin activity of these two *Amaranthus* vegetable. However, lower income people in less developed countries comparatively evaded from this fetal disease especially from prostate and breast cancer [22] but they live on nothing but else rice and weedy vegetables including *Amaranthus*. Therefore, we were inspired from this finding and designed this study to evaluate antioxidant, lectin, antimicrobial as well as anticancer activity of these two *Amaranthus* species using the rodent animal (mouse) as diseases model containing EAC cells. Laboratory mouse is widely used as model organism, sharing 99 % of their genes with human being along with very similar biochemical organization and serve as a safe and reliable platform to manipulate a complex disease process in a manner impossible to perform in patients [23, 24]. Laboratory mouse is being used for long time in different *in vivo* experiment to screen anticancer agent from plant sources [25, 26]. Therefore, this study was carried out to evaluate the medicinal property of AH and AL in terms of antioxidant, anticancer as well as antimicrobial activity in the literature.

## Methods

### Chemicals and reagents

DPPH and Trypan blue dye, DAPI, Methanol (Sigma, USA); BHT and DMSO (Merck, Germany); M-MLV reverse transcriptase, 1^st^ strand buffer, dNTPs, and primer of oligo (dT), p53, Bax, caspase-3, Bcl-2 and β-actin (Tiangen Biotech, Beijing, China).

### Plant materials

Fresh, young AL as well as mature AH plant with ripen seed were collected from the field of the surrounding area of Rajshahi, Bangladesh in January 2014. The identities of both the plant were authenticated by the taxonomist at the Botany Department of the University of Rajshahi, Bangladesh. A voucher specimen (Accession number: 1447) was deposited at the national herbarium Dhaka, Bangladesh.

### Determination of antioxidant activity

#### Preparation of plant extract

Both of the sample were sterilized properly using standard technique and shade dried at room temperature for 15 days and then grinded into fine powder. The resultant powder was added with 100 % methanol and kept in a shaking incubator (160 rpm) for 24 h at 37 °C followed by centrifugation at 8000 rpm for 15 min. The resultant pellets were remixed with the same percentage of methanol and kept at shaking incubator for 12 h. The collected supernatants were filtered through filter paper and then allowing the filtrate to evaporate using a rotary evaporator for several times. The concentrated methanol extracts of AL and AH was stored at −20 °C for DPPH radical scavenging assay.

### DPPH radical scavenging assay

Antioxidant activity of both the plant extract was evaluated using DPPH radical scavenging assay [27]. An estimated 2.4 mg of DPPH was dissolved in 100 ml methanol and diluted with methanol to obtain an absorbance of 0.98 (± 0.03) at 517 nm using the spectrophotometer (Thermo scientific, China). An aliquot of 100 μl extract of both sample at the concentration of 25, 50 and 100 μg/ml were added in 3 ml DPPH solution, separately. Butylated hydroxytoluene (BHT) was used as standard. The mixtures were incubated in dark at room temperature for 20 min and the absorbance was recorded at 517 nm. DPPH radical scavenging activity was calculated using the following formula:

$$ \mathrm{Scavenging}\ \mathrm{effect}\ \left(\%\right) = \left[\left(\mathrm{Control}\ \mathrm{absorbance}\right)\ \hbox{--}\ \left(\mathrm{sample}\ \mathrm{absorbance}\right)/\left(\mathrm{control}\ \mathrm{absorbance}\right)\right] \times 100 $$

### Determination of lectin activity

The lectin activity of crud *Amaranthus* extracts was determined by hemmaglutination assay [28]. Briefly, the stem of AL (5 g) and seed of AH (5 g) were grinded with 1 % sodium chloride saline (3 ml/g) using mortar and spatula and then centrifuged at 12000 rpm for 5 min for 2 times. In a 96-well microtiter U plate, 50 μl test sample was placed in the first well and then serially diluted into the successive wells with phosphate buffered saline (PBS), pH 7.4. An aliquot of 50 μl of 2 % mouse blood suspension was added in each wall. PBS alone was added as control. The titer plate was then kept at 37 °C for 30 min and observed the agglutination of blood. Hemagglutination activity was assessed as agglutination of blood at lowest concentration of extract.

### Determination of anticancer activity

#### Preparation of plant extract

The water extract was used to evaluate the anticancer potential of *Amaranthus* species. In brief, the shade dried stem of AL and seed of AH were blended by a blander to get fine powder. Then 25, 50 and 100 μg of resultant powder were mixed with 1 ml deionized double distilled water (dH_2_O) and centrifuged at 12000 rpm for 5 min.

### Experimental animal, ethics statement and cancer cell inoculation and treatment

A total of forty two mature female Swiss albino mice (25-30 g) were purchased from the Department of Pharmacy of Jahangernagar University, Dhaka, Bangladesh. The animals were kept in the animal house of the Department of Biochemistry and Molecular Biology, University of Rajshahi, Bangladesh. The methodology used in the current research work along with handling of experimental animal was approved by the Institutional Animal, Medical Ethics, Biosafety and Biosecurity Committee (IAMEBBC) for Experimentations on Animal, Human, Microbes and Living Natural Sources (license no: 225/320-IAMEBBC/IBSc), Institute of Biological Sciences, University of Rajshahi, Bangladesh.

EAC cells used in this study were kindly provided by Protein and Enzyme Laboratory, Department of Biochemistry and Molecular Biology, University of Rajshahi, Bangladesh. Mice were injected with EAC cells by successive transplantation of 6 × 10^6^ cells/mouse in peritoneal cavity by needle aspiration with a volume of 0.2 ml in PBS.

Mice injected with EAC cells on day zero were divided into two major groups namely treated and control group. Treated group was then divided into three subgroups (each group contain six animals) for each *Amaranthus* species as: group 1, group 2 and group 3, received 25, 50 and 100 μg/ml/day/mouse of test extracts, respectively after 24 h of EAC cells injection. Animals of the control group were received only 2 % DMSO solution at 5 ml/kg/mouse/day.

### Determination of cell growth inhibition

The measurement of *in vivo* cancer growth inhibition was conducted by the method previously described by Sur et al. [29]. At the end of six days treatment, the animals were anesthetized using diethyl-ether and then intraperitoneal EAC cells were diluted with normal saline (0.98 %) followed by harvesting with needle. Viable EAC cells were counted on hemocytometer using trypan blue dye with light microscope (optika, Italy). The cell growth inhibition was calculated using the following formula:

$$ \%\ \mathrm{Cell}\ \mathrm{growth}\ \mathrm{inhibition} = \left(1\hbox{-} \mathrm{T}\mathrm{w}/\mathrm{C}\mathrm{w}\right) \times 100 $$

Where,

Tw = Mean number of EAC cells in the treated mice

Cw = mean number of EAC cells in the control mice.

### Apoptosis assessment by DAPI staining

Collected EAC cells (1 ml) from each group of mice were centrifuged at 1200 rpm for 2 min. The plate was then washed with PBS for each time after centrifugation at 1200 rpm for 2 min for three times. The resultant cells were then incubated with 5 μl DAPI staining solution in dark for 10 min with subsequent adding of PBS to the DAPI containing pellet and then centrifuged at 1200 rpm for 2 min. Finally, 200 μL PBS was added to the pellet and 10 μl of the supernatant was taken on a microscopic slide and observed the morphological changes of cancer cells under the fluorescence microscope (XDS-2FL, Optika, Italy).

### RNA isolation, cDNA synthesis and PCR amplification of p53, Bax, Bcl-2 and caspase-3

Total RNA was isolated from the EAC cells of both control and treated (100 μg/ml) mice using TIAGEN reagent kit according to the manufacturer’s protocol. The quality of RNA was checked by 1 % agarose gel electrophoresis, stained with 10 μg/ml ethidium bromide and visualized using gel documentation system (Alphaimager mini, Taiwan). The concentration and purity of isolated RNA was assessed by spectrometry at 260 and 280 nm. Properly isolated RNA was converted to cDNA using reverse transcription master mix (20 μl), containing 2 μl oligo (dT), 1 μl M-MLV reverse transcriptase, 2 μl dNTPs, 4 μl 5× 1^st^ strand buffer and 3 μ total RNA sample and 8 μl dH_2_O. The primer sequences used in the study are shown in Table 1. The thermal cycler (Gene Atlas 482, Japan) program for amplification reactions was set at 95 °C for 3 min, 95 °C for 1 min and 1 min for 52 °C (35 cycles) followed by 72 °C for 1 min, and 72 °C for 10 min and eventually hold at 20 °C. Relative expression of p53, Bax, Bcl-2 and caspase-3 mRNA was measured by comparing with the expression of β-actin mRNA.

**Table 1:** The primers used for PCR amplification

Gene	Primer sequence
β-actin	Forward : 5′-GAGACCTTCAACACCCCAGC-3′
	Reverse : 5′-ATGTCACGCACGATTTCCC-3′
p53	Forward : 5′-CACAAAAACAGGTTAAACCCAG-3′
	Reverse : 5′-AGCACATAGGAGGCAGAGAC-3′
Caspase-3	Forward : 5’ - GCAGCAAACCTCAGGGAAAC-3′
	Reverse : 5′- GGTTTCCCTGAGGTTTGCTG-3′
Bax	Forward : 5′-CCTGCTTCTTTCTTCATCGG-3′
	Reverse : 5′-AGGTGCCTGGACTCTTGGGT -3′
Bcl-2	Forward : 5′- GGCTGGGATGCTTTGTG-3′
	Reverse : 5′- GAGCAGTGCCTTCAGAGACAGC-3′

### Determination of Antibacterial activity

#### Extraction of total protein content for antibacterial assay

Freshly collected stem of AL and seed AH were blended by mortar and spatula with Tris–HCl buffer. Then the resulted material was homogenized with Tris–HCl buffer (1 ml/10 mg plant materials) as well as β-mercapto ethanol (1 μl) then vortexes for proper mixing. The homogenized mixture was then centrifuged at 10,000 rpm for 20 min and the supernatant was stored at 4 °C.

#### Disc diffusion assays

Disc diffusion assay was carried out to measure the bacterial susceptibility to *Amaranthus* extract. The bacterial cultures used in the study were two Gram positive bacteria including *Staphylococcus aureus* (ATCC 29213) and *Bacillus subtilis* (ATCC 441) and three Gram negative bacteria including *Escherichia coli (*ATCC 25922)*, Pseudomonas aeruginosa* (ATCC 27853) and *Salmonella typhi*. All the test microorganisms were kindly provided by Microbiology Laboratory, Department of Genetic Engineering and Biotechnology, University of Rajshahi, Bangladesh. Sterile paper discs (6 mm, Whatman, Maidstone, UK) were impregnated with both the plant extract (50 μg/disc). The test organisms (100 μl) were inoculated on the surface of solid agar medium and incubated one hour before placing the paper discs. Then the agar plates were incubated at 37 °C for 24 h. Kanamycin (15 μg/disc) was used as positive control.

### Statistical analysis

Statistical analyses for the assessment of antioxidant and growth inhibitory activity of *Amaranthus* extract in comparison with control was performed using one way ANOVA and student’s *t*-test method. Data are expressed as mean ± SD (*n* = 3) for antioxidant study. Data are expressed as mean ± SD (*n*= 6) for anticancer study. The significance was set at *P* <0.05 and *P* <0.01.

## Results

### Antioxidant activity by DPPH radical scavenging assay

DPPH radical scavenging activity of the extract of two *Amaranthus* species along with BHT standard is shown in Fig. 1. The methanol extracts of AL and AH exhibited dose dependent scavenging activity against DPPH free radicals. The seed extract of AH demonstrated higher free radical scavenging rate, exhibiting IC_50_ value of 28 ± 1.8 μg/ml (Table 2) over than the stem extract of AL (with IC_50_ value of 93 ± 2.44 μg/ml). However, the scavenging activity of both plant extract was less significant (*P* <0.01) in comparison with BHT standard (IC_50_ 12 ± 0.5 μg/ml).

**Fig. 1:** DPPH radical scavenging activity of methanol extracts were isolated from the stem of AL and seed of AH. BHT was used as positive control. Each value represents a mean ± SD (*n* = 3)

**Table 2:** Half maximal inhibitory concentration (IC_50_) of the AL and AH along with BHT standard

Samples	IC_50_ values (μg/ml)
*A. lividus*	93 ± 2.44
*A. hybridus*	28 ± 1.8
BHT	12 ± 0.5**

Each value is represented as mean ± SD (*n* = 3), significance was set at *P* <0.01 (**) with respect to BHT standard

### Assessment of lectin activity

The hemagglutination activity of stem extract of AL and seed extract of AH is shown in Fig. 2. Both of the *Amaranthus* species demonstrated concentration dependant hemagglutination activity on mice blood. According to the data, the seed extract of AH shows hemagglutination activity at 1.565 μg/wall, while the stem extract of AL required comparatively higher concentration (3.125 μg/wall) to agglutinate the blood. However, negative control did not show hemagglutination activity at any concentration.

**Fig. 2:** Hemagglutination activity of crud extract of the stem of AL and seed of AH. Stem of AL shows hemagglutination activity on mice blood at 3.125 μg/wall, but in case of AH this activity was at 1.565 μg/wall. The control titer-plate did not show hemagglutination at any concentration of PBS

### Anticancer activity

#### Growth inhibitory activity of *Amaranthus* extract on EAC cells

The anti-proliferative activity of two *Amaranthus* species is shown in Fig. 3 and Table 3. The percentage of EAC cells growth inhibition as a consequence of six days administration of *Amaranthus* extract is shown in Fig. 3b. Hemocytometer counting of EAC cells using trypan blue dye was shown to decrease the viability of EAC cells considerably in all treated groups in comparison with control. According to the data presented in Fig. 3b, seed extract of AH has relatively higher growth inhibitory activity and exhibiting 14, 26 and 45 % growth inhibition at 25, 50 and 100 μg/ml, respectively over than stem extract of AL (12, 21 and 43 %, respectively) at the same concentration (Fig. 3b).

**Fig. 3:** Growth inhibitory activity of *Amaranthus* extract at different concentration on EAC cells. **a** Hemocytometer counting of EAC cells collected from both control and treated groups was determined using trypan blue dye after six days of EAC cells injection. **b** Percentage of growth inhibition of EAC cells on each concentrations of *Amaranthus* extract (counting the percentage in treated groups by considering zero cell death in control group). Each value represents a mean ± SD (*n* = 6 )

**Table 3:** Growth inhibitory activity of *Amaranthus* extract on EAC cells by hemocytometer counting using trypan blue dye

Plants	Average count of EAC cells per cell of hemocytometer (out of 16 cells)			
	Control	25 μg	50 μg	100 μg
*A. lividus*	32 ± 0.52	28 ± 0.56	25 ± 0.38*	18 ± 0.33**
*A. hybridus*	32 ± 0.52	27.37 ± 0.5	23.37 ± 0.58*	17.25 ± 0.41**

Each value is represented as mean ± SD (*n* = 6), significance was set at *P* <0.05 (*) and *P* <0.01 (**) with respect to control

### Detection of apoptotic EAC cell by DAPI staining

To observe the morphological changes of apoptotic EAC cells after the ending of six days treatment, DAPI staining was performed. Figure 4a reveals the marked feature of apoptosis in all the treated groups when compared with round shaped and less brightly stained control cells. Whereas the apoptotic cells or ongoing apoptotic cells exhibited bright blue color with condense chromatin. Reversely to the normal cells, the apoptotic cells exhibited characteristic apoptotic changes such as membrane blebbing, cell shrinkage, chromatin condensation, nuclear fragmentation and aggregation of apoptotic bodies etc (Fig. 4a). The average number of apoptotic cells/ slide is shown in Fig. 4b. Animals treated with both the *Amaranthus* extract at 50 and 100 μg/ml show significantly (at *P* <0.05 and *P* <0.01, respectively) elevated number of apoptotic cells in comparison with control mice.

**Fig. 4:** Detection of apoptotic cells using DAPI staining after six days of treatment. **a** Treatment was started after 24 h of EAC cells injection, at the concentration of 25, 50 and 100 μg/ml. Marked apoptotic features such as membrane blebbing, cell shrinkage, chromatin condensation, aggregation of apoptotic bodies and brightly stained nucleus under blue fluorescence etc were observed in the treated groups, in contrast to round shaped and less brightly stained control cells. **b** Number of apoptotic cells per side was estimated by counting apoptotic cells in five different fields. Each value represents as mean ± SD (*n* = 3). Significance was set at *P* <0.05 (*) and *P* <0.01 (**) with respect to control

### The contribution of p53, caspase-3, Bax and Bcl-2 in apoptosis

To observe the expression pattern of several vital apoptotic markers such as p53, Bax, Bcl-2 and caspase-3, gene amplification study was conducted. The result from gene amplification study demonstrated that the animals treated with the extracts at 100 μg/ml showed up-regulation of p53, Bax and caspase-3 mRNA when compared with their respective controls (Fig. 5b). Considerably lower expression of Bcl-2 mRNA in 100 μg/ml treated mice was also observed, which indicates mitochondria mediated apoptosis of EAC cells.

**Fig. 5:** Apoptotic changes of EAC cells induced by *Amaranthus* extract were found to mediated by mitochondrial pathway: **a** Isolated total RNA exhibited two separate bands as 28S and 18S. **b** The animals treated with *Amaranthus* extract at 100 μg/ml for six days exhibited relatively up-regulation of p53, Bax and caspase-3 and showing bright and bolder band in comparison with control. While the expression of Bcl-2 mRNA was decreased considerably when compared with the control. Beta-actin was used as standard

### Assessment of antimicrobial activity

The bacterial susceptibility to the crud protein of AL and AH is shown in Fig. 6. Both of the plant extract exhibited negligible inhibition of bacterial growth in comparison with the positive control (both at *P* <0.05 and *P* <0.01). Among the bacterial species *E. coli* shows comparatively higher sensitivity to the *Amaranthus* extract (8.6 *±* 0.79 mm for AL extract and 9.4 *±* 0.61 mm for AH extract).

**Fig. 6:** Bacterial susceptibility to the crud protein of two *Amaranthus* species was conducted using disc diffusion assay. Antimicrobial activity was determined by measuring the zone of inhibition in millimeter (mm). Kanamycin (15 μg/disc) was used as positive control. Each value represents a mean ± SD (*n* = 3). Significance was set at *P* <0.05 (*) and *P* <0.01 (**) with respect to control

## Discussion

Nowadays, scientific communities and pharmaceutical companies are aim to find out bioactive phytochemicals exerting health-promoting benefits in a non toxic way. Combination of chemotherapeutic agents with naturally occurring tumor active compounds such as polyphenols would be better able to overcome mechanisms of drug resistance. Excessive ROS levels in normal cells has been reported to be involved in various aspects of carcinogenesis by altering cellular signaling and gene expression pattern [4, 30]. Plant derived dietary compounds play anticancer role either by increasing ROS level in cancer cells, resulting induction of programmed cell death or counter-regulating elevated ROS level in normal cells by antioxidant mechanism [31]. The antioxidant molecules can balance the ROS level either by neutralizing and producing less active, longer-lived and less dangerous new free radicals or destroy them by reacting with the reactive radicals directly.

In the present study, we have investigated antioxidant, lectin, antimicrobial and anticancer activity of stem and seed extract of two vegetable species of *Amaranthus* using different staining and gene expression technique. Stem extract of AL and seed extract of AH at different concentrations exhibited strong scavenging activity against DPPH stable radicals (Fig. 1). A number of *Amaranthus* species have been proven previously to possess considerable antioxidant capacity. However, our current findings show that methanol extract of AL and AH exhibited comparatively higher antioxidant potential than those of other species of *Amaranthus* even the other extracts of these species [32, 33].

The strong anticancer activity in this study would be the result of lectin activity present in the *Amaranthus* extract. Lectins are a class of glycoprotein present mainly in plant especially in seed in abundant quantity and having carbohydrate binding capacity. Lectin activity in plant sample is usually determined by hemagglutination assay. The elevated hemagglutination activity of seed extract over stem extract is also supported by a number of studies which show that higher lectin content in seed sample over than the other parts of the plant [34]. Higher lectin activity of seed sample also supports the comparative higher anti-proliferative outcome of seed extract over the stem extract in the current study (Fig. 3). Since, lectin has been reported to possess remarkable anti-antitumor activity, exerting apoptotic role by preferential binding to cancer cell membranes with subsequent cytotoxicity [35]. Lectin also exhibits growth inhibitory activity by altering the cell cycle and inducing non-apoptotic G1-phase accumulation mechanisms, G2/M phase cell cycle arrest and apoptosis [36]. Therefore, plant lectin can be considered as a potential agent for combinational therapy against a range of cancer cell lines. Nevertheless, the crude protein of two vegetable species of *Amaranthus* did not show considerable antimicrobial activity against tested pathogenic bacteria (Fig. 6). Such insignificant antimicrobial activity of AH and AL has also been documented previously in case of other *Amaranthus* species [37].

Apoptosis is an ideal way of cell death by which the body selectively eliminates unnecessary cells or unhealthy cells in a series of sequential events without affecting surrounding normal cell. Inhibition of apoptosis is the critical early event in tumor development, which allows the cell to proliferate abnormally and leading to the development of cancer [38]. Therefore, induction of apoptosis is considered as a central strategy and a useful indicator for almost every type’s cancer treatment and prevention. Trypan blue dye and DAPI staining study exhibited the growth inhibitory activity of *Amaranthus* extracts on EAC cells by induction of apoptosis. The number of viable cells were found to be decreased by around 45 % (Fig. 3) at 100 μg/ml, indicating significant growth inhibitory activity of *Amaranthus* extracts on cancer cells (Fig. 3b). The dose dependant depletion of EAC cells is considered to be the result of induction of apoptosis pathway which modulates cells death [39]. DAPI staining clearly demonstrated the critical morphological features of apoptosis including membrane blebbing, cell shrinkage, chromosome condensation, nuclear fragmentation and aggregation of apoptotic bodies etc. Membrane blebbing and cell shrinkage are considered to be the key morphological alterations of early apoptotic cells. Whereas DNA fragmentation and aggregation of apoptotic bodies are the end products of apoptosis and would be the result of catalytic activities of executioner caspases (caspases-3 and caspases-7).

Apoptosis involves a series of sequential protein-protein interactions which is basically regulated by the ratio of anti-apoptotic and pro-apoptotic proteins belonging to Bcl-2 family. Anti-apoptotic Bcl-2-like proteins (e.g. Bcl-2, Bcl-xL, Bcl-w, Mcl-1 and A1/Bfl-1) down-regulate apoptosis by protecting mitochondrial membrane potential, whereas pro-apoptotic Bax-like proteins (e.g. Bax, Bak and Bok/Mtd) up-regulate apoptosis by creating pore on the mitochondrial membrane. It has been well reported that plant derived phytochemicals induce oxidative DNA damage in cancer cells by producing elevated level of ROS [31] which in turn induces up-regulation of p53, the critical regulator of mitochondria mediated apoptosis, inducing apoptosis by up-regulating some critical apoptotic modulators such as puma, Noxa and Bax [40, 41]. Activated Bax then translocates to and inserts into the mitochondrial outer membrane [42] with subsequent releasing of cytochrome *c* (Cyt *c*) in the cytosol. Mitochondrial Cyt *c* in cytosol binds with its binding partner Apaf-1 which in turn binds with procaspase-9 and forms a large wheel like multi-protein complex “apoptosome” [43]. The activated caspase-9 then cleaves the proenzyme form of the effector caspases such as caspase-3, caspase-6 and caspase-7 [44]. Caspase-3 is the key effectors caspase in apoptosis which acts by restricted proteolysis of important cellular proteins mainly the structural proteins such as cytokeratins, PARP and nuclear protein NuMA, resulting cell death [45]. Therefore, we have evaluated the expression pattern of these apoptotic markers in *Amaranthus* treated animals and in the control counterparts in this study. The up-regulation of p53, Bax and caspase-3 mRNA as well as down-regulation of Bcl-2 mRNA in treated mice indicated the induction of mitochondria mediated apoptosis of EAC cells. The apparent apoptotic features in DAPI staining EAC cells of treated mice also support the alteration of genetic expression indicating apoptotic death of cancer cells. The outcomes of our current study are in accord with a number of observations which demonstrated that the bioactive phytochemicals generate elevated level ROS which in turn induces mitochondria mediated apoptosis by up-regulating the expression of p53 and pro-apoptotic proteins (Bax) and down-regulating the expression of anti-apoptotic proteins (Bcl-2) follwed by activating caspases-3 [15, 46]. Therefore, it could be postulated that the phytochemicals (lectins, polyphenols, flavonoids) present in *Amaranthus* extract would produce elevated level of ROS which in turn induces over-expression of p53 and induction of mitochondria mediated apoptosis of EAC cells.

Here, the anticancer activity of the stem extract of AL and seed extract of AH on EAC cells could be attributed to the presence of a variety of bioactive phytochemicals. Till date we do not know what bioactive compound played the key anti-proliferative role on EAC cells. Another limitation of this study is that we did not carry out anti-proliferative study on *in vitro* cell line. Furthermore, detection of specific bioactive phyto-ingredients demonstrating anticancer effect will be of great therapeutic value. Nevertheless the current study provides the proof of strong evidence that *Amaranthus* possesses potent anticancer property with great health benefit to common people and can be considered as a potential target for future research.

## Conclusion

In conclusion, our data suggest that the treatment of EAC cells with lectin rich *Amaranthus* extract inhibited the growth of cancer cells by induction of apoptosis. The gene expression pattern in *Amaranthus* treated mice clearly exhibited that the stem extract of Al and seed extract of AH induced mitochondria mediated apoptosis of EAC cells. However, the complete mechanisms underlying the therapeutic effects of the extract such as cytotoxicity need to be investigated as an approach for the development of effective combinational therapy against a range of cancer cell line.

## Abbreviations

%: percentage; AH: *Amaranthus hybridus*; AL: *Amaranthus lividus*; ANOVA: one way analysis of variance; BHT: Butylated hydroxytoluene; DAPI: 4΄,6-diamidino-2-phenylindole; DMSO: Dimethyl sulfoxide; EAC: Ehrlich’s ascites carcinoma; mg: milligramme; mL: milliliter; nm: nanometer; PBS: phosphate buffered saline; ROS: Reactive oxygen species; rpm: rotation per minutes; Tris–HCl: Tris- hydrochloric acid; μL: microliter
